# Addition of 5-fluorouracil to first-line induction chemotherapy with docetaxel and cisplatin before concurrent chemoradiotherapy does not improve survival in locoregionally advanced nasopharyngeal carcinoma

**DOI:** 10.18632/oncotarget.20017

**Published:** 2017-08-07

**Authors:** Wang Fangzheng, Jiang Chuner, Wang Lei, Yan Fengqin, Ye Zhimin, Sun Quanquan, Liu Tongxin, Xu Min, Wu Peng, Long Bin, Rihito Aizawa, Masoto Sakamoto, Fu Zhenfu

**Affiliations:** ^1^ Department of Radiation Oncology, Zhejiang Cancer Hospital, Zhejiang Hangzhou, 310022, People’s Republic of China; ^2^ Zhejiang Key Laboratory of Radiation Oncology, Zhejiang Hangzhou, 310022, People’s Republic of China; ^3^ Department of Radiology, Japanese Red Cross Fukui Hospital, Fukui, 918-8501 Japan; ^4^ Department of Breast Tumor Surgery, Zhejiang Cancer Hospital, Zhejiang Hangzhou, 310022, People’s Republic of China; ^5^ Department of Physics, Zhejiang Cancer Hospital, Zhejiang Hangzhou, 310022, People’s Republic of China; ^6^ Department of Pathology, Zhejiang Cancer Hospital, Zhejiang Hangzhou, 310022, People’s Republic of China; ^7^ Department of Nuclear Medicine, Zhejiang Cancer Hospital, Zhejiang Hangzhou, 310022, People’s Republic of China; ^8^ Department of Radiation Oncology and Image-applied Therapy, Graduate School of Medicine, Kyoto University, 606-8507, Kyoto, Japan

**Keywords:** nasopharyngeal carcinoma, induction chemotherapy, concurrent chemoradiotherapy, toxicity, prognosis

## Abstract

Although a multicenter, randomized study indicated that induction chemotherapy (IC) with docetaxel/cisplatin/fluorouracil (TPF) before concurrent chemoradiotherapy (CCRT) improves survival outcomes, it remains unclear whether TPF is the best IC regimen for treating locoregionally advanced nasopharyngeal carcinoma (NPC). Our aim was to compare the efficacy and toxicities of TPF vs. docetaxel/cisplatin (TP) IC followed by CCRT in patients with locoregionally advanced NPC. One hundred thirty-two patients with locoregionally advanced NPC received 21-day cycles of IC with either TPF or TP. Both were followed by intensity-modulated radiotherapy concurrent with the cisplatin treatment every 3 weeks. Three-year rates of locoregional relapse-free survival, distant metastasis-free survival, progression-free survival, and overall survival were respectively 96.4%, 87.7%, 86.0%, and 94.7% for patients in the TPF arm patients and 90.3%, 91.9%, 85.2%, and 92.0% for patients in the TP arm. There were no differences in survival between the two arms. Multivariate analysis revealed the IC regimen was not an independent prognostic factor for any survival outcome. However, patients in the TP arm experienced fewer grade 3/4 toxicities. In sum, IC with docetaxel and cisplatin is associated with similar efficacy and less toxicity than the TPF regimen. Addition of fluorouracil to docetaxel plus cisplatin IC is therefore not recommended for patients with locoregionally advanced NPC.

## INTRODUCTION

Nasopharyngeal carcinoma (NPC) is a common head and neck cancer in Southern China, Malaysia, and Singapore [1]. Radiotherapy (RT), the main treatment for non-disseminated NPC, results in 5-year overall survival (OS) rates of 90–100% in stage I–II and 60–85% in stage III-IVB patients [2, 3]. However, over 70% of NPC patients are diagnosed with locoregionally advanced diseases, and survival outcomes are poor in these patients [4]. The advent of intensity-modulated radiotherapy (IMRT), improvements in radiological techniques, and the application of concurrent chemotherapy have improved locoregional control, and distant failure is now typically the main cause of mortality [5–8]. The efficacies of induction chemotherapy (IC), concurrent chemoradiotherapy (CCRT), and adjuvant chemotherapy (AC) have been compared. CCRT is a standard treatment for patients with locoregionally advanced NPC and results in better survival outcomes than RT alone [9–11]. Because few patients completed all three treatment cycles, AC was not associated with therapeutic gain in these patients [12]. The combination of IC followed by CCRT has therefore been studied more extensively. Phase II studies revealed that IC together with CCRT increased locoregional control rates for locoregionally advanced NPC [13, 14]. OuYang *et al.* found that adding IC to CCRT treatment reduced distant metastasis and improved OS [15]. Additional research is needed to examine the efficacy of treatments that combine IC and CCRT.

It remains unclear which IC regimen is most effective in patients with locoregionally advanced NPC. IC with cisplatin and fluorouracil (PF) has been widely used as a first-line regimen in NPC patients for many years. However, PF did not improve survival compared to CCRT alone [16, 17]. Taxanes, which are microtubule inhibitors, inhibit cell division. Several randomized phase III trials reported that the addition of taxane to IC regimens with cisplatin alone (TP) or with cisplatin and 5-fluorouracil (TPF) improved treatment outcomes in patients with locoregionally advanced head and neck squamous cell cancer [18–20]. A recent phase 3 multicenter, randomized trial published in Lancet Oncology indicated that the addition of docetaxel, cisplatin, and 5-flurouracil (TPF) to CCRT improved OS, failure-free survival, and distant metastases-free survival (DMFS) rates in patients with locoregionally advanced NPC compared to CCRT alone [21]. Kong *et al.* also recently demonstrated that the addition of TPF-based IC to CCRT improved survival outcomes in locoregionally advanced NPC patients in comparison with historical data [22].

Although TPF-based IC followed by CCRT results in better survival outcomes than CCRT alone, it remains unclear whether TPF is the best IC regimen for NPC patients. Here, we conducted a phase II study to compare the efficacy and tolerability of TPF vs. TP IC regimens followed by concurrent chemotherapy and IMRT for patients with locoregional advanced NPC.

## RESULTS

### Patient basic characteristics and therapy adherence

One hundred thirty-two eligible patients with locoregionally advanced NPC treated between January 2012 and January 2014 were randomly assigned to the TPF arm (*n* = 57) or the TP arm (*n* = 75). Basic patient demographic information and tumor characteristics are summarized in Table 1. Patient and tumor characteristics were similar between the two treatment arms.

**Table 1:** Basic patient demographic information and tumor characteristics

Characteristic	TPF regimen	TP regimen	*X*^*2*^	*p*
	*N* = 57	*N* = 75		
Gender			0.025	0.874
Male	41	53		
Female	16	22		
Age (years)			0.710	0.400
Range	19–63	22–70		
Median	47	49		
< 50	39	46		
≥ 50	18	29		
WHO pathology			1.712	0.425
Type I	3	1		
Type II	2	3		
Type III	52	71		
ECOG performance status			0.022	0.882
0	45	60		
1	12	15		
T stage*			2.560	0.465
T1	1	2		
T2	10	21		
T3	31	32		
T4	15	20		
N stage*			1.980	0.372
N0	0	0		
N1	7	11		
N2	40	57		
N3	10	7		
Clinical stage*			0.094	0.760
III	35	48		
IV	22	27		
Comorbidity			0.386	0.534
No	48	60		
Yes	9	15		

Abbreviations: WHO, World Health Organization; ECOG, Eastern Cooperative Oncology Group, *The 7th AJCC/UICC staging system.

### Disease response

After IC, 18 patients (31.6%) displayed complete remission (CR), 37 (64.9%) displayed partial remission (PR), and 2 (3.5%) displayed stable disease (SD) for nasopharyngeal tumors in the TPF arm, while 23 (40.4%), 49 (65.3%), and 3 (4.0%) TP arm patients displayed CR, PR, and SD, respectively. For cervical metastatic lymph nodes, CR, PR, and SD rates were 36.8% (21/57), 61.4% (35/57), and 1.8% (1/57) in TPF arm patients and 38.7% (29/75), 58.7% (44/75), 2.6% (2/75) in TP arm patients, respectively. After the completion of IMRT, CR rates for nasopharyngeal tumors and neck metastatic lymph nodes were 91.2% and 94.7% in TPF arm patients and 92.0% and 93.3% in TP arm patients, respectively. No statistically significant differences in disease responses to treatment were found between two arms (Table 3).

**Table 2:** Therapy details for the two arms

Treatment	TPF regimen	TP regimen	*p*
Cycle of IC			0.928
1	3	3	
2	39	53	
3	15	19	
Cycle of CC			0.659
0	8	15	
1	26	31	
2	23	29	
AC			0.019
No	7	22	
Yes	50	53	

Abbreviations: IC, induction chemotherapy; CC, concurrent chemotherapy; AC, adjuvant chemotherapy; TP, docetaxel/cisplatin; TPF, docetaxel/cisplatin/fluorouracil.

**Table 3:** Tumor responses to treatment in the two arms

Response	Nasopharyngeal tumor		*p*	Neck lymph node		*p*
	TPF (*n*, %)	TP (*n*, %)		TPF (*n*, %)	TP (*n*, %)	
IC						
CR	18 (31.6)	23 (40.4)	0.985	21 (36.8)	29 (38.7)	0.910
PR	37 (64.9)	49 (65.3)		35 (61.4)	44 (58.7)	
SD	2 (3.5)	3 (4.0)		1 (1.8)	2 (2.6)	
CCRT						
CR	52 (91.2)	69 (92.0)	0.874	54 (94.7)	70 (93.3)	0.738
PR	5 (8.8)	6 (8.0)		3 (5.3)	5 (6.7)	

Abbreviations: IC, induction chemotherapy; CCRT, concurrent chemoradiotherapy; CR, complete remission; PR, partial remission; SD, stable disease; TP, docetaxel/cisplatin; TPF, docetaxel/cisplatin/fluorouracil.

### Survival outcomes

Survival was assessed for all patients with locoregionally advanced NPC in follow-ups conducted after a median of 47 months (range, 13–60 months). The estimated locoregional relapse-free survival (LR-RFS), distant metastasis-free survival (DMFS), progression-free survival (PFS), and overall survival (OS) rates were 93.0%, 90.1%, 85.5%, and 93.2%, respectively, after 3 years (Figure 1).

**Figure 1:** Kaplan-Meier estimates of survival in 132 NPC patients

There were no statistically significant differences in LR-RFS, DMFS, PFS, or OS between the two arms (3-year LR-RFS: 96.4% vs. 90.3%, respectively, *p* = 0.199, Figure 2A; 3-year DMFS: 87.7% vs. 91.9%, respectively, *p* = 0.554, Figure 2B; 3-year PFS: 86.0% vs. 85.2%, respectively, *p*=0.835, Figure 2C; 3-year OS: 94.7% vs. 92%, respectively, Figure 2D).

**Figure 2:** Kaplan-Meier estimates of survival outcomes in TPF and TP arm NPC patients

All patients finished a full course of radical IMRT and received 1-3 cycles of IC. One hundred nine (82.6%) patients received CC and 103 (78.0%) received AC. Differences in treatments between the two arms are listed in Table 2.

### Analysis of treatment failure

Twenty-two patients experienced treatment failure. Among these patients, 6 (1 in the TPF arm and 5 in the TP arm) developed locoregional relapse, 6 (2 in the TPF arm and 4 in the TP arm) had locoregional relapse and distant metastases, and 10 (6 in the TPF arm and 4 in the TP arm) experienced distant relapse. Treatment failure modes in these patients are summarized in Table 4. The median time to failure was 19 months (range, 8 to 39 months) for TPF arm patients versus 15 months (range, 6 to 55 months) for TP arm patients.

**Table 4:** Treatment failure details

Failure mode	TPF	TP	*p*
	*N* = 57	*N* = 75	
Locoregional	1	5	0.374
Locoregional and distant	2	4	
Distant	6	4	
No failure	48	62	

### Prognostic factors

Patient age, patient gender, clinical stage, adjusted tumor (T) and lymph node (N) stage, comorbidities, and IC regimen were examined as potential prognostic factors. Factors that influenced survival outcomes were identified and their prognostic roles evaluated in univariate and multivariate analyses. Univariate analysis revealed that 3-year DMFS, PFS, and OS had higher predictive value in stage III NPC patients than in stage IVA-B patients (3-year DMFS: 95.2% vs. 81.3%, *p* = 0.005; PFS: 92.8% vs. 73.0%, *p* = 0.001; OS: 96.4% vs. 87.8%, *p* = 0.004), and age was associated with LR-RFS (Table 5). Multivariate analysis indicated that age was an independent prognostic factor of LR-RFS (*p* = 0.035), and clinical stage was an independent predictor of DMFS (*p* = 0.010), PFS (*p* = 0.002), and OS (*p* = 0.011) (Table 6).

**Table 5:** Factors predictive of survival outcomes in 132 NPC patients identified via univariate analysis

Characteristics	*n*	LRRFS (%)	*p*	DMFS (%)	*p*	PFS (%)	*p*	OS (%)	*p*
Age			0.024		0.349		0.980		0.672
< 50	85	96.3		88.1		85.7		94.1	
≥ 50	47	87.0		93.6		85.1		91.5	
Gender			0.705		0.727		0.743		0.746
Male	94	93.4		88.3		85.1		92.5	
Female	38	91.9		94.6		86.5		94.7	
T stage			0.121		0.422		0.138		0.440
T1–2	34	97.0		91.2		91.2		94.1	
T3–4	98	91.6		89.7		83.5		92.9	
N stage			0.256		0.356		0.939		0.560
N0–1	18	88.9		100		88.9		94.4	
N2–3	114	93.6		88.5		83.5		93.0	
Clinical stage			0.082		0.005		0.001		0.004
III	83	96.4		95.2		92.8		96.4	
IVA/B	49	86.8		81.3		73.0		87.8	
Comorbidity			0.503		0.219		0.267		0.898
No	108	93.3		88.9		84.2		93.5	
Yes	24	91.3		95.8		91.5		91.7	
IC regimen			0.199		0.554		0.835		0.434
TPF	57	96.4		87.7		86.0		94.7	
TP	75	90.3		91.9		85.2		92.0	

Abbreviations: LRRFS, locoregional relapse-free survival; DMFS, distant metastases-free survival; PFS, progression-free survival; OS, overall survival; IC, induction chemotherapy; TP, docetaxel/cisplatin; TPF, docetaxel/cisplatin/fluorouracil.

**Table 6:** Effects of prognostic factors on survival outcomes in multivariate analysis

Endpoint	Characteristic	HR	95% CI	*p*-value
OS	III vs. IV	0.184	0.050–0.679	0.011
PFS	III vs. IV	0.242	0.098–0.594	0.002
LRRFS	< 50 vs. ≥ 50 years	0.274	0.083–0.911	0.035
DMFS	III vs. IV	0.247	0.086–0.711	0.002

Abbreviations: OS, overall survival; PFS, progression-free survival; LRRFS, locoregional recurrence-free survival; DMFS, distant metastasis-free survival.

### Safety and toxicity

The most commonly observed complications included hematologic and non-hematologic side effects. During IC treatment (Table 7), grade 3 or higher leukocytopenia and neutropenia were reported in 33 (57.9%) and 44 (77.2%) of TPF arm patients, respectively, and in 14 (24.6%) and 17 (22.7%) of TP arm patients, respectively; these complications were more common in TPF arm patients (*p* < 0.001). Additionally, more TPF arm patients suffered mucositis and diarrhea than did TP arm patients (17 vs. 7, *p* = 0.002; 19 vs. 5, *p* < 0.001). The frequency of other toxicities did not differ between patients in the two arms.

**Table 7:** Adverse events during IC in the two arms

Adverse events	TPF arm					TP arm					*Z*	*p*
	0	1	2	3	4	0	1	2	3	4		
Hematologic												
Leukocytopenia	1	4	19	29	4	8	22	31	10	4	–4.874	< 0.001
Neutropenia	1	6	8	20	22	14	15	29	12	5	–5.758	< 0.001
Anemia	39	14	3	1	0	51	15	7	2	0	–0.233	0.816
Thrombocytopenia	45	2	9	1	0	60	5	10	0	0	–0.278	0.781
Liver function	27	24	5	1	0	43	25	7	0	0	–1.066	0.286
Renal function	56	1	0	0	0	75	0	0	0	0	–1,147	0.251
Non-hematologic												
Mucositis	40	10	5	2	0	68	5	2	0	0	–3.062	0.002
Dermatitis	52	5	0	0	0	69	6	0	0	0	–0.158	0.874
Diarrhea	38	15	3	1	0	70	3	2	0	0	–3.850	< 0.001
Nausea/vomiting	45	7	4	1	0	67	5	2	1	0	–1.644	0.100

Abbreviations: IC, induction chemotherapy.

Incidences of acute adverse events by type and grade after CCRT are shown in Table 8. Frequencies of hematologic events, RT-related mucositis, and dermatitis did not differ between the two arms.

**Table 8:** Adverse events after CCRT in the two arms

Adverse events	TPF arm					TP arm					*Z*	*p*
	0	1	2	3	4	0	1	2	3	4		
Hematologic												
Leukocytopenia	15	20	18	4	0	16	30	17	12	0	–0.676	0.499
Neutropenia	14	14	19	8	2	24	29	12	7	3	–1.839	0.066
Anemia	43	10	4	0	0	51	18	6	0	0	–0.886	0.375
Thrombocytopenia	42	6	6	3	0	61	5	6	2	1	–1.000	0.371
Liver function	46	10	1	0	0	69	6	0	0	0	–1.935	0.053
Renal function	56	1	0	0	0	75	0	0	0	0	–1.147	0.251
Non-hematologic												
Mucositis	0	26	28	3	0	0	35	36	4	0	–0.106	0.915
Dermatitis	0	53	3	1	0	0	70	5	0	0	–0.105	0.916
Diarrhea	51	3	2	1	0	70	3	2	0	0	–0.815	0.415
Nausea/vomiting	49	7	1	0	0	64	6	4	1	0	–0.215	0.830

Abbreviations: CCRT, concurrent chemoradiotherapy.

## DISCUSSION

In the present study, we found that both docetaxel/cisplatin IC before IMRT with concurrent cisplatin-based chemotherapy (TP arm) and docetaxel/cisplatin/fluorouracil IC before CCRT (TPF arm) result in similar survival outcomes. Additionally, incidences of leucocypenia, neutropenia, mucositis, and diarrhea (hematologic toxicities) were lower in TP arm patients than in TPF arm patients. Thus, the addition of fluorouracil to treatments with docetaxel plus cisplatin may not improve survival in patients with locoregionally advanced NPC.

Three-year LR-RFS, DMFS, PFS, and OS rates did not differ between the two treatment arms. Among the potential prognostic factors examined, we found that age was an independent prognostic factor of LR-RFS and clinical stage was an independent predictor of DMFS, PFS, and OS.

Since the TAX 323 and 324 studies established TPF as the most effective IC treatment for improving survival outcomes in head and neck cancer [18, 19], a growing number of studies have examined IC regimens that include taxanes. Recently, Ma *et al.* reported that three cycles of TPF IC before CCRT significantly improved survival outcomes, with 3-year OS, failure-free survival, and DMFS rates of 92%, 80%, and 90%, respectively [21]. Kong *et al.* reported 3-year OS, PFS, DMFS, and LRFS rates of 94.8%, 78.2%, 90.5%, and 93.9%, respectively, for a TPF-based IC regimen in the treatment of locoregionally advanced NPC [22]. Hassan *et al.* found that the addition of TP-based IC to CCRT resulted in good local control of locoregionally advanced NPC with a manageable toxicity profile [23]. In a randomized phase II trial, Hui *et al.* demonstrated that 2 cycles of TP IC before CRT improved 3-year OS compared to CRT alone (94.1% vs. 67.7%) [24]. In another phase II trial of TP together with CCRT, Zhong *et al.* observed 3-year OS and PFS rates of 94.1% and 72.7%, respectively [25]. While treatment with docetaxel and cisplatin with or without fluorouracil has resulted in excellent survival outcomes as a first-line IC for locoregionally advanced NPC, few studies have compared the efficacy and safety of TP versus TPF followed by CCRT in these patients. We therefore conducted the present phase II study to compare the efficacy and tolerability of TPF versus TP with concurrent chemotherapy and IMRT in these patients. Our results demonstrated that either TPF or TP in combination with CCRT yielded similar survival outcomes.

Hematologic and non-hematologic toxicities were the most commonly observed complications during the treatment period. Incidences of grade 3 or higher leukocytopenia and neutropenia were lower in patients who received TP treatment than in those who received TPF (24.6% vs. 57.9% and 22.7% vs. 77.2%, respectively). The incidences of hematologic toxicities observed here in TPF-treated patients are similar to those observed in previous studies (ranging from 55–83%) [18, 19, 22, 26]. All patients in this study received prophylaxis leukocyte therapy using recombinant granulocyte colony-stimulating factor (GCFS), and patients who experienced grade 3/4 leukocytopenia and neutropenia during IC and could therefore continue with chemotherapy without delay. Non-hematological side effects, such as mucositis, dermatitis, diarrhea, and nausea/vomiting, were mild to moderate. Incidences of mucositis and diarrhea were lower in TP arm patients than in TPF arm patients (9.3% and 22.7% and 6.7% vs. 33.3%, respectively). Similar percentages of patients in the two treatment arms completed more than 2 cycles of IC.

In conclusion, our results suggest that TPF and TP IC regimens before IMRT plus concurrent chemotherapy yield similar disease responses and LR-RFS, DMFS, PFS, and OS rates in locoregionally advanced NPC, while TP results in a better toxicity profile. However, further randomized, controlled, multicenter phase III clinical trials are needed to assess the efficacy and toxicity of TP IC regimens.

## MATERIALS AND METHODS

### Patients and pretreatment

The patients enrolled in this study were hospitalized between January 2012 and January 2014 in the Department of Radiation Oncology, Zhejiang Cancer Hospital. Eligible patients met the following criteria: (i) histologically confirmed NPC; (ii) aged 18 to 70 years; (iii) stage III/IVA-B at diagnosis (American Joint Committee on Cancer staging system, 7th edition); (v) adequate bone marrow, liver and renal function; (vi) no previous anti-cancer treatment.

The exclusion criteria were as follows: aged 70 years or older; previously received RT, chemotherapy, or surgery for tumors; had distant metastases before treatment; were pregnant; history of other malignancy; severe comorbidities. This prospective randomized study was approved by the medical ethics committee of Zhejiang Cancer Hospital. All patients signed written informed consent before participating in this research.

Patients underwent a pretreatment evaluation that included collection of complete medical history, physical examination, hematology and biochemistry profiles, chest radiographs, sonography of the abdomen, bone scan, magnetic response imaging of the nasopharynx, and nosopharyngoscope. All patients were staged according to 2010 AJCC staging system. Tumor histology was classified according to the World Health Organization classifications.

Treatment details are shown in Figure 3. A total of 158 newly diagnosed locoregionally advanced NPC patients were randomly assigned to receive either the TPF or TP IC regimen before CCRT. The efficacy and toxicity of the two IC regimens in combination with CCRT were evaluated in 132 of these patients.

**Figure 3:** Trial profile

### Treatment schemes

#### Radiation therapy

All patients were immobilized in a supine position with thermoplastic masks. Computed tomography scans with intravenous contrast (2.5 mm slices from the head to 2 cm below the sternoclavicular joints) were performed for planning purposes. Target volumes were delineated according to the recommendations of the International Commission on Radiation Units and Measurements CTV delineation protocol for head and neck malignancies [27, 28]. The delineation of NPC target volumes during the IMRT treatment was performed as described previously [29, 30]. Gross tumor volume (GTV) referred to the extent of the tumor in clinical and imaging examinations. The extent of the primary tumor, including metastatic retropharyngeal lymph nodes, was defined as GTVnx, and the metastatic lymph nodes of the neck as GTVnd.

CTV was defined individually according to GTV and potential regions at risk surrounding the nasopharyngeal cavity. CTV for GTVnx included CTVnx for the high-risk CTV and CTV1 when invasion was present. CTVnx was defined as GTVnx plus a 7-mm margin that encompassed the nasopharyngeal mucosa plus 5 mm submucosal volume. For CTV1, the potentially involved anatomic regions were the entire nasopharyngeal cavity, the anterior one- to two-thirds of the clivus (when invasion was present, the whole clivus was covered), the skull base, the pterygoid plates, the parapharyngeal space, the inferior sphenoid sinus (the entire sphenoid sinus was be covered for stage T3 and T4 NPC), the posterior one-quarter to one-third of the nasal cavity, and the maxillary sinus. High-risk nodes included level Ib nodes in patients with metastatic lymph nodes in level IIa, and any lymph nodes in drainage pathways containing metastatic lymph nodes. Low-risk areas for prophylactic neck irradiation areas were referred as CTV2. These low-risk areas included levels IV and Vb without metastatic cervical lymph nodes.

PTV was constructed automatically based on each volume with an additional 3-mm margin in three dimensions to account for set-up variability. All PTVs, including PGTVnx, PTVnx, PTV1, and PTV2, were not delineated outside of the skin surface. Critical normal structures, including the brainstem, spinal cord, parotid glands, optic nerves, chiasm, lens, eyeballs, temporal lobes, temporomandibular joints, mandible, and hypophysis, were contoured and set as OARs during optimization.

All patients underwent radical IMRT with simultaneous integrated boost technique using 6 MV photons. The prescribed radiation dose was 70 or 72 Gy to PGTVnx, 66–70 Gy to PGTVnd, 62–66 Gy to PTVnx, 60–63 Gy to PTV1, and 51–54 Gy to PTV2, delivered in 30 or 33 fractions. Radiation was delivered once daily, five fractions per week, over 6–6.5 weeks for IMRT planning. The dose to OAR was limited based on the RTOG 0225 protocol.

### Chemotherapy regimens

All eligible patients were given one to three cycles of platinum-based induction chemotherapy at 3-week intervals. The TPF IC regimen consisted of docetaxel 60 mg/m^2^/day on day 1, cisplatin 25 mg/m^2^/day on days 1–3, and 5-fluorouracil 500 mg/m^2^/day on days 1–3; the TP IC regiment consisted of docetaxel 60 mg/m^2^/day on day 1 and cisplatin 25 mg/m^2^/day on days 1–3.

NPC patients in this study also underwent ≥ 1 cycle of concurrent chemotherapy with cisplatin (80 mg/m^2^) divided over 3 days. One hundred three patients received 2–3 courses of adjuvant chemotherapy with an FP (cisplatin 25 mg/m^2^/day on days 1–3 and 5-fluorouracil 500 mg/m^2^/day on days 1–3) regimen 3 weeks after RT.

### Patient evaluation and follow-up

Tumor responses were assessed three times: after the completion of induction chemotherapy, at the end of IMRT, and 3 months after radiation, which was based on MRI and nasopharynx fiberscope according to Response Evaluation Criteria for Solid Tumors criteria. Systemic chemotherapy adverse effects were graded using the National Cancer Institute Common Toxicity Criteria (NCI CTCAE, version 3.0), whereas RT-induced toxicities were scored according to the Acute and Late Radiation Morbidity Scoring Criteria of the Radiation Therapy Oncology Group (RTOG).

All the subjects underwent weekly examinations for treatment response and toxicities during radiation therapy. Patient followed-ups occurred every 3 months for the first 2 years, every 6 months from the third to the fifth year, and annually thereafter. Each follow-up included careful examination of the nasopharynx and neck nodes by an experienced doctor, MRI scan of the nasopharynx, nasopharynx fiberscope, chest computed tomography radiograph, and ultrasound of abdomen performed 3 months after the completion of RT and every 6–12 months thereafter. Additional examinations were performed as needed to evaluate local relapse or distant metastasis.

### Statistical analysis

The end points of this study included LRRFS, DMFS, PFS, OS, and acute toxicities from IC and CCRT. OS was calculated from the date of enrollment to the date of death or the last follow-up. LRRFS, DMFS, and PFS were calculated from the date of enrollment to the date of locoregional relapse, distant metastasis occurrence, diagnosed evidence of disease progression, or the last follow-up. After recurrence or metastasis, patients were given salvage therapy as determined by their physicians.

Descriptive statistics were used to compare the patients’ characteristics, treatment adherence, tumor response, and patterns of failure between the two arms. Two independent sample non-parametric tests were used to compared acute toxicity between the two arms. Survival curves were generated using the Kaplan-Meier method. The curves were compared using log-rank tests. Multivariate analysis was performed using Cox regression models to identify significant prognostic factors. Hazard ratios (HRs) and 95% confidence intervals (CIs) were calculated for each prognostic factor. IBM SPSS Statistics version 19.0 was used for all data analysis. *P* < 0.05 was considered statistically significant.
